The article "Combined Association of Low-Density Lipoprotein Cholesterol Levels and Systolic Blood Pressure to the Outcome of Intracerebral Hemorrhage: Data from the China Stroke Center Alliance" was retracted in 2024. Reasons: signs of a paper mill; suspected computer-generated content; unreliable results or conclusions; missing or withdrawn patient consent.

# Combined Association of Low-Density Lipoprotein Cholesterol Levels and Systolic Blood Pressure to the Outcome of Intracerebral Hemorrhage: Data from the China Stroke Center Alliance

**DOI:** 10.1155/2022/6206315

**Published:** 2022-06-18

**Authors:** Yarong Ding, Yu Wang, Liping Liu, Hongqiu Gu, Kaixuan Yang, Zixiao Li, Xingquan Zhao

**Affiliations:** ^1^Department of Neurology, Beijing Tiantan Hospital, Capital Medical University, Beijing, China; ^2^China National Clinical Research Center for Neurological Diseases, Beijing, China; ^3^Department of Neurology, Beijing Luhe Hospital, Capital Medical University, Beijing, China; ^4^Department of Neurology, Beijing Hospital, National Center of Gerontology, Beijing, China; ^5^Research Unit of Artificial Intelligence in Cerebrovascular Disease, Chinese Academy of Medical Sciences, Beijing, China; ^6^Department of Epidemiology and Health Statistics, School of Public Health, Capital Medical University, Beijing, China; ^7^Beijing Municipal Key Laboratory of Clinical Epidemiology, Beijing, China

## Abstract

Limited data were available about the combined impact of systolic blood pressure (SBP) and low-density lipoprotein cholesterol (LDL-C) levels on intracerebral hemorrhage (ICH) prognosis. The objective of this study is to explore whether the relationship between LDL-C and ICH outcomes was modified by SBP levels in a Chinese population. From August 1, 2015, to July 31, 2019, 75,443 ICH patients enrolled from the Chinese Stroke Center Alliance program were included in our study. Patients were divided into LDL-C levels of <70 mg/dL, 70-100 mg/dL, and ≥100 mmol/L. SBP was stratified as <140 mmHg, 140-180 mmHg, and ≥180 mmHg. The primary outcome was the occurrence of hematoma expansion (HE), and the second outcome was in-hospital mortality. Correlation between LDL-C levels and SBP on ICH outcomes were assessed by logistic regression. 6,116 (8.1%) and 1,576 (2.1%) patients suffered HE and in-hospital mortality. Compared with the ≥100 mg/dL group, patients with LDL-C concentrations under 70 mg/dL had a 19% and 24% increase in the relative risk of HE (crude OR 1.19, 95% CI 1.11-1.28) and in-hospital mortality (crude OR 1.24, 95% CI 1.08-1.42). When SBP was added as a stratification variable, the above-mentioned association was attenuated in patients under a threshold SBP of 140 mmHg (*P* > 0.05). However, no statistical interaction was detected between SBP and LDL-C levels. Lower LDL-C levels (<70 mg/dL) are related to a higher risk of HE and in-hospital mortality confined to ICH patients with elevated SBP (≥140 mmHg).

## 1. Introduction

Intracerebral hemorrhage (ICH) has significant high morbidity and mortality [1–3]. Interventional trials, involving intensive antihypertensive treatment [4], hypoglycemic therapy [5], hemostatic agents [6, 7], and hematoma evacuation [8, 9], achieved only marginally therapeutic efficacy. As interest in multifactorial interventions is increasing, integrated approaches to the management of ICH are urgently needed.

Elevated blood pressure (BP), especially systolic BP (SBP), is the cornerstone of ICH prevention as is closely related to the occurrence of hematoma expansion (HE) and subsequent poor prognosis [10]. Meanwhile, growing attention has been paid to the effect of low-density lipoprotein cholesterol (LDL-C) on ICH prognosis [11–13]. In the series of China Stroke Center Alliance (CSCA) studies, we found that in acute ICH patients, lower LDL-C levels are related to a high risk of HE and mortality [14]. Researches regarding the joint effects of SBP and LDL-C on atherosclerotic cardiovascular risk showed an additive, even synergetic association [15–17]. While limited data were available about the combined impact of SBP and LDL-C levels on ICH prognosis. It is worth noting that one observational research indicated that the proportional risk of cerebral hemorrhage associated with lower LDL-C was confined to patients with elevated BP [18].

Therefore, the purpose of our study was to investigate whether the association between LDL-C and ICH prognosis was modified by SBP levels in a Chinese population.

## 2. Materials and Methods

### 2.1. Study Population

The CSCA program was initiated by the Chinese Stroke Association in June 2015 to establish a national, hospital-based stroke care quality assessment and improvement platform, the protocol of which has been previously reported [19]. From August 1, 2015, to July 31, 2019, 1,006,798 stroke or transit ischemic attack patients within 7 days from the onset were recruited consecutively from 1,576 hospitals. A total of 85,705 spontaneous ICH patients were selected for the initial assessment in our study. Among all the recruited patients, 4,152 individuals were excluded due to incomplete data on baseline SBP or LDL-C levels, 154 individuals without data on HE, and 293 individuals with incomplete in-hospital mortality data were also excluded. Besides, 5,663 individuals with unclear time from symptom onset to hospital arrival were excluded. Eventually, 75,443 patients were included in this final analysis (Figure 1). Baseline characteristics between included and excluded ICH patients are shown in Table S1; the clinical features of which were similar in general.

The study was conducted in compliance with the Helsinki Declaration and approved by the central Institutional Review Board at Beijing Tiantan Hospital.

### 2.2. LDL-C, SBP, and Other Baseline Covariates

Laboratory variables were collected within 24 hours after admission to each subcenter. LDL-C levels were categorized into three groups regarding the 2018 American Heart Association guidelines for the management of cholesterol: <70 mg/dL, 70-100 mg/dL, and ≥100 mg/dL [20].

Three BP readings were recorded separately in the supine position after at least two-minute resting by trained nurses at baseline, and the average of the three measurements was regarded as the admission BP. Admission SBP was then classified into three categories based on the 2018 European Society of Hypertension as <140 mmHg, 140-180 mmHg, and ≥180 mmHg [21].

Other baseline characteristics including demographic information, body mass index (BMI), smoking and drinking history, medical and medication history, Glasgow coma scale (GCS) score on admission, and time from symptom onset to arrival were also extracted.

### 2.3. Outcomes

The primary outcome was HE event, and the second outcome was in-hospital mortality. A cranial CT scan was obtained in the emergency department and repeated after admission. Hematoma volume was estimated using the ABC/2 method by two experienced neurologists [22]. According to the radiographic criteria, HE was diagnosed by follow-up image as the intraparenchymal hematoma increased >33% or an absolute increment of >6 mL from initial hematoma [23].

### 2.4. Statistical Analysis

Data were presented as mean ± standard deviation (SD) or median (interquartile range, IQR) for continuous variables and count (percentage) for categorical variables. The ANOVA or nonparametric Kruskal-Wallis test and the chi-squared test were used in the comparison of baseline variables.

The independent correlation between LDL-C, SBP, and ICH prognosis was assessed by odds ratios (ORs) and 95% confidence interval (CI) using logistic regression. The subgroups with the highest LDL-C (≥100 mg/dL) and SBP levels (≥180 mmHg) were used as the reference. Model 1 was corrected for age and sex. Model 2 was further adjusted for BMI (<25.0 or ≥25.0 kg/m^2^), systolic and diastolic BP, smoking, drinking, hypertension, diabetes mellitus, previous ICH, medication history (including prior use of the antiplatelet, anticoagulant, antihypertensive agent, and stains), and creatinine. Since the GCS score was only recorded in 39,216 (52.0%) patients, model 3 was performed as a sensitivity analysis in those with complete GCS score information on admission. Besides, to assess whether a differential correlation between lower LDL-C with HE or in-hospital mortality is observed in different SBP categories, an interaction term (LDL-C × SBP, both as a polytomous variable) was added among all the included patients as well as patients admitted within 24 h of symptom onset.

Differences were considered to be significant at *P* < 0.05. Analyses were performed using the SAS software (version 9.4; SAS Institute, Cary, NC, USA).

## 3. Results

75,443 patients were finally enrolled in our study; 6,116 (8.1%) and 1,576 (2.1%) of them were identified as HE and in-hospital mortality, separately. Among them, the lowest LDL-C group (<70 mg/dL) together with the highest SBP group (≥180 mmHg) tended to have more events. The prevalence of adverse outcomes according to LDL-C levels across SBP subgroups is shown in Figure 2.

### 3.1. Baseline Characteristics

Significant differences were found in age, sex, BMI, BP, behavior history, previous history, medication history, in-hospital treatment, creatinine, and GCS score on admission among LDL-C groups. Baseline characteristics and ICH prognosis according to LDL-C categories are shown in Table 1.

### 3.2. Independent Association of LDL-C and SBP Levels for ICH Outcomes

Lower LDL-C levels had a significant correlation with ICH outcomes in the univariate analysis (*P* < 0.001). Compared with the ≥100 mg/dL group, patients with LDL-C concentrations under 70 mg/dL had a 19% and 24% increase in the relative risk of HE (OR 1.19, 95% CI 1.11-1.28) and in-hospital mortality (OR 1.24, 95% CI 1.08-1.42). In the multivariate analysis, similar results were obtained after adjusting for potential covariates in model 1 and 2. The adjusted ORs of HE were 1.17 (95% CI 1.09-1.26) for LDL − C levels < 70 mg/dL, 1.02 (95% CI 0.96-1.08) for LDL-C levels of 70 mg/dL to 100 mg/dL, and 1.0 (reference) for LDL − C levels ≥ 100 mg/dL in model 2. Correspondingly, the adjusted ORs of in-hospital mortality were 1.16 (95% CI 1.01-1.33), 0.96 (95% CI 0.86-1.08), and 1.0 (reference) among the three LDL-C groups from low to high. However, increasing mortality risk with lower LDL-C levels (<70 mg/dL) was not pronounced when further adjusted for admission GCS score in the sensitivity analysis.

The fully adjusted ORs of the lowest SBP group (<140 mmHg) were 0.82 (95% CI 0.73-0.93) and 0.74 (95% CI 0.60-0.90) for HE and in-hospital mortality, respectively. Additional detailed information was given in Table 2.

### 3.3. Combined Association of LDL-C and SBP to ICH Outcomes

When examining the association of LDL-C with ICH outcomes across SBP categories, it was noteworthy that no statistical significance was obtained in those with SBP under 140 mmHg, irrespective of LDL-C concentration (*P* > 0.05). While for those with SBP between 140 mmHg and 180 mmHg and SBP above 180 mmHg, lower LDL-C levels (<70 mg/dL) conferred a 1.23-fold, 1.16-fold greater likelihood of HE presence (*P* < 0.001, Table 3). When it comes to in-hospital mortality, its significant correlation with lower LDL-C levels diminished among the highest SBP category (≥180 mmHg). In multivariate analyses, the results were essentially unaltered in both model 1 and model 2. While after further adjustment for admission GCS score in model 3, the association became nonsignificant between lower LDL-C levels and adverse outcomes among ICH patients with normal SBP. There was, however, no apparent interaction detected between LDL-C and SBP with either HE (*P* = 0.649) or in-hospital mortality (*P* = 0.667).

To differentiate the effect of time from symptom onset to admission, additional sensitivity analyses were performed among the 60,024 patients admitted within 24 h of symptom onset. In these analyses, consistent with the overall population, lower LDL-C level (<70 mg/dL) was accompanied by a higher risk of HE and in-hospital mortality, particularly in individuals with a baseline SBP above 140 mmHg (Figure 3).

## 4. Discussion

We provided evidence of ICH risk stratification regarding LDL-C concentrations across SBP categories in acute ICH patients. Those with LDL − C < 70 mg/dL conferred a higher risk of HE and in-hospital mortality compared to patients with LDL − C ≥ 100 mg/dL. When SBP was added as a stratification variable, it was noteworthy that the above-mentioned association was attenuated in patients under a threshold SBP of 140 mmHg. Patients admitted within 24 h of symptom onset presented robust consistent results. However, no statistical interaction was detected between SBP and LDL-C levels. Our results indicated that the adverse outcome occurs commonly in the high-risk ICH patients, those with lower LDL-C levels and uncontrolled BP, for whom intensive control of SBP is recommended.

Although with the popular belief of lipid-lowering goal towards “the lower, the better” in atherosclerotic cardiovascular disease [24], appropriate LDL-C levels are still a matter of debate when weighing atherosclerosis and bleeding in acute ICH. Observational studies with small sample size demonstrated that lower LDL-C levels were independently related to HE in ICH patients [25, 26]. What is more, recent studies suggested that lower LDL-C levels carried an increased hazard of mortality [12, 25]. Of the 75,443 ICH patients enrolled in our study, the fully adjusted OR of HE for the lowest versus the highest LDL-C group was 1.22 (95% CI 1.10-1.35). When it comes to in-hospital mortality, full adjustment with admission GCS score attenuated the significant association with LDL-C. In the series of CSCA studies, the correlation between LDL-C and adverse events weakened with the aggravation of ICH [14].

Research about the strength and shape of the joint effects of SBP and LDL-C levels on hemorrhagic risk was limited. Data from the China Kadoorie Biobank prospective study showed that lowering LDL-C by 1 mmol/L increased the risk of ICH by about one-seventh, irrespective of baseline BP level [11], while another Korean observational study suggested that the inverse association between serum cholesterol and hemorrhagic stroke was restricted to hypertensive [18]. The results of our study added to the evidence that the bleeding risk associated with lower LDL-C (<70 mg/dL) in acute ICH patients with elevated SBP (≥140 mmHg). BP in the hyperacute phase of ICH was strongly related to adverse outcomes [10]; we thus performed a sensitivity analysis among patients admitted within 24 h of symptom onset which yielded identical results to the overall population. However, no apparent modification effect of SBP subgroups was discovered in the relationship between LDL-C and ICH prognosis. Our investigation suggested that acute ICH patients with lower LDL-C and elevated BP are more susceptible to HE and ensuing mortality; simultaneous control of these two factors may have therapeutic potential.

Hypertension is a well-recognized hazard factor for adverse outcomes in ICH patients, and intensive BP reduction was associated with reduced HE and improved functional outcomes [10]. Furthermore, cholesterol is important for the integrity of vessel walls. While in the pathological state of ICH with poor BP control, decreased cholesterol levels could lead to the fragility of cerebrovascular endothelium [27], promote the necrosis of arterial smooth muscle cells [28], inhibit platelet aggregation [29], affect erythrocyte osmotic fragility [30], and eventually cause bleeding [31]. A combined but noninteractive effect of circulating LDL-C and SBP levels on ICH outcomes was observed in our study. Intensive control of SBP to 140 mmHg is rational and necessary, especially for acute ICH patients with lower LDL-C levels.

Our study confirmed and extended the results of our previous investigation by further adding SBP categories; lower LDL-C levels are related to an increased hazard of HE and in-hospital mortality in patients with poorly-controlled BP. Nonetheless, there are still some limitations. First, hematoma volume at baseline and follow-up were unaccessible, and the determination of HE relied on subcenters. Meanwhile, the time from symptom onset to CT scans was unobtainable in the CSCA program. Secondly, our study included patients who underwent surgery, which may cause selection bias. While the statistical significance remained after excluding 7,511 patients taken operation (data was not shown). Thirdly, despite no statistical significance being reached between lower LDL-C and poor prognosis in ICH patients with SBP controlled under 140 mmHg, these results should be interpreted with caution as the exact value of ORs were all above 1.00. Besides, further analysis focused on different hypertension grades (grade 1 and 2) compared with normotension was needed given the wide SBP thresholds in our study.

## 5. Conclusions

A combined but noninteractive effect of LDL-C and SBP levels on ICH outcomes was observed in our study. Lower LDL-C levels (<70 mg/dL) are associated with a higher risk of HE and in-hospital mortality confined to ICH individuals with elevated SBP (≥140 mmHg).

## Figures and Tables

**Figure 1:** Flow chart for selection of study participants. TIA: transit ischemic attack; CSCA: Chinese Stroke Center Alliance; LDL-C: low-density lipoprotein cholesterol; SBP: systolic blood pressure; ICH: intracerebral hemorrhage.

**Figure 2:** Prevalence of (a) hematoma expansion and (b) in-hospital mortality according to LDL-C levels across systolic blood pressure subgroups. LDL-C: low-density lipoprotein cholesterol.

**Figure 3:** Association of LDL-C with HE or in-hospital mortality across SBP categories among patients admitted within 24 h of symptom onset^‡^. LDL-C: low-density lipoprotein cholesterol; HE: hematoma expansion; SBP: systolic blood pressure. *P* = 0.747 for HE; *P* = 0.604 for in-hospital mortality. ^‡^60,024 (79.6%) patients were admitted within 24 h of symptom onset.

**Table 1:** Characteristics of enrolled participants according to LDL-C levels.

Variables	Total	LDL-C levels			*P* value
		<70 mg/dL	70-100 mg/dL	≥100 mg/dL	
*n* (%)	75433	11899 (15.8)	24952 (33.1)	38592 (51.2)	
Age, years	63.0 ± 12.8	64.2 ± 12.8	63.6 ± 12.9	62.2 ± 12.8	<0.001
Male, *n* (%)	47079 (62.4)	8306 (69.8)	16134 (64.7)	22639 (58.7)	<0.001
BMI, kg/m^2^	23.9 ± 4.2	23.5 ± 3.7	23.7 ± 3.7	24.1 ± 4.7	<0.001
SBP, mmHg	164.7 ± 27.9	162.4 ± 28.2	164.3 ± 27.7	165.6 ± 27.9	<0.001
DBP, mmHg	95.3 ± 16.8	93.5 ± 16.4	94.8 ± 16.5	96.2 ± 16.9	<0.001
Current smoker, *n* (%)	14905 (19.8)	2561 (21.5)	5088 (20.4)	7256 (18.8)	<0.001
Current alcoholic, *n* (%)	18373 (24.4)	3101 (26.1)	6049 (24.2)	9223 (23.9)	<0.001
Previous history, *n* (%)					
Hypertension	53939 (71.5)	8377 (70.4)	17562 (70.4)	28000 (72.6)	<0.001
Diabetes mellitus	7200 (9.5)	1301 (10.9)	2107 (8.4)	3792 (9.8)	<0.001
Dyslipidemia	3108 (4.1)	416 (3.5)	764 (3.1)	1928 (5.0)	<0.001
Heart failure	347 (0.5)	83 (0.7)	114 (0.5)	150 (0.4)	<0.001
Previous ICH	12877 (17.1)	2190 (18.4)	4174 (16.7)	6513 (16.9)	<0.001
Previous ischemic stroke	21333 (28.3)	3875 (32.6)	6994 (28.0)	10464 (27.1)	<0.001
Medication history, *n* (%)					
Antiplatelet	5296 (7.0)	1265 (10.6)	1731 (6.9)	2300 (6.0)	<0.001
Anticoagulant	1332 (1.8)	267 (2.2)	386 (1.5)	679 (1.8)	<0.001
Antihypertensive agent	35928 (47.6)	5765 (48.4)	11642 (46.7)	18521 (48.0)	<0.001
Statins	4380 (5.8)	1017 (8.5)	1356 (5.4)	2007 (5.2)	<0.001
In-hospital treatment, *n* (%)					
Hematoma evacuation	7511 (10.0)	1408 (11.8)	2457 (9.8)	3646 (9.4)	<0.001
Antihypertensive agent	54635 (72.4)	8254 (69.4)	17899 (71.7)	28482 (73.8)	<0.001
Statins	18310 (24.3)	2693 (22.6)	5312 (21.3)	10305 (26.7)	<0.001
Creatinine, *μ*mol/L	67.6 (55.0, 84.3)	67.0 (54.6, 83.1)	67.0 (55.0, 82.0)	68.0 (55.0, 86.0)	<0.001
GCS score on admission^∗^	14.0 (8.0, 15.0)	13.0 (7.0, 15.0)	14.0 (8.0, 15.0)	14.0 (9.0, 15.0)	<0.001
Time from onset to arrival, hours	3.8 (1.5, 21.0)	3.5 (1.5, 18.3)	3.8 (1.6, 20.5)	3.9 (1.5, 22.0)	0.918
Hematoma expansion, *n* (%)	6116 (8.1)	1102 (9.3)	1977 (7.9)	3037 (7.9)	<0.001
In-hospital mortality, *n* (%)	1576 (2.1)	296 (2.5)	500 (2.0)	780 (2.0)	0.004

Values are (%) for categorical variables and mean ± SD or median (IQR) for continuous variables. SD: standard deviation; LDL-C: low-density lipoprotein cholesterol; BMI: body mass index; SBP: systolic blood pressure; DBP: diastolic blood pressure; ICH: intracerebral hemorrhage; GCS: Glasgow coma scale. ^∗^GCS score on admission was evaluated in 39,216 (52.0%) patients.

**Table 2:** Odds ratios of ICH outcomes for LDL-C and SBP levels measured at baseline.

	Variables	Case (%)	Univariate analysis	Multivariate analysis		
				Model 1	Model 2	Model 3
LDL-C	Hematoma expansion					
	<70 mg/dL	1102 (9.26)	1.19 (1.11, 1.28)	1.19 (1.11, 1.28)	1.17 (1.09, 1.26)	1.22 (1.10, 1.35)
	70-100 mg/dL	1977 (7.92)	1.01 (0.95, 1.07)	1.00 (0.95, 1.07)	1.02 (0.96, 1.08)	1.02 (0.94, 1.11)
	≥100 mg/dL	3037 (7.87)	Ref.	Ref.	Ref.	Ref.
	In-hospital mortality					
	<70 mg/dL	296 (2.49)	1.24 (1.08, 1.42)	1.16 (1.01, 1.33)	1.16 (1.01, 1.33)	0.91 (0.76, 1.08)
	70-100 mg/dL	500 (2.00)	0.99 (0.88, 1.11)	0.95 (0.85, 1.06)	0.96 (0.86, 1.08)	0.87 (0.75, 1.00)
	≥100 mg/dL	780 (2.02)	Ref.	Ref.	Ref.	Ref.
SBP	Hematoma expansion					
	<140 mmHg	1055 (8.33)	0.95 (0.87, 1.02)	0.95 (0.88, 1.02)	0.90 (0.83, 0.98)	0.82 (0.73, 0.93)
	140-180 mmHg	3074 (7.66)	0.86 (0.81, 0.91)	0.86 (0.81, 0.91)	0.83 (0.78, 0.88)	0.78 (0.72, 0.85)
	≥180 mmHg	1987 (8.78)	Ref.	Ref.	Ref.	Ref.
	In-hospital mortality					
	<140 mmHg	213 (1.68)	0.51 (0.44, 0.60)	0.52 (0.45, 0.61)	0.51 (0.43, 0.59)	0.74 (0.60, 0.90)
	140-180 mmHg	633 (1.58)	0.48 (0.43, 0.54)	0.47 (0.43, 0.53)	0.47 (0.42, 0.52)	0.67 (0.58, 0.76)
	≥180 mmHg	730 (3.22)	Ref.	Ref.	Ref.	Ref.

Data are OR (95% CI) unless otherwise stated. Model 1 adjusted for age and sex. Model 2 adjusted for variables in model 1 plus body mass index (<25.0 or ≥25.0 kg/m^2^), systolic blood pressure, diastolic blood pressure, smoking status, drinking status, hypertension, diabetes mellitus, previous ICH, medication history (including prior use of antiplatelet, anticoagulant, antihypertensive agent, and stains), and creatinine. Model 3 adjusted for variables in model 2 plus GCS score on admission as a sensitivity analysis.

**Table 3:** Association between LDL-C and ICH outcomes in different blood pressure levels among all the included patients.

SBP	LDL-C levels	Case (%)	Univariate analysis	Multivariate analysis		
				Model 1	Model 2	Model 3
Hematoma expansion						
<140 mmHg	<70 mg/dL	214 (9.18)	1.18 (0.99, 1.39)	1.17 (0.99, 1.38)	1.14 (0.96, 1.35)	1.16 (0.90, 1.49)
	70-100 mg/dL	364 (8.45)	1.07 (0.93, 1.24)	1.07 (0.93, 1.23)	1.07 (0.93, 1.24)	0.98 (0.79, 1.22)
	≥100 mg/dL	477 (7.92)	Ref.	Ref.	Ref.	Ref.
140-180 mmHg	<70 mg/dL	563 (8.93)	1.23 (1.11, 1.36)	1.23 (1.11, 1.36)	1.20 (1.08, 1.33)	1.33 (1.14, 1.54)
	70-100 mg/dL	996 (7.51)	1.02 (0.94, 1.11)	1.02 (0.94, 1.11)	1.04 (0.96, 1.13)	1.13 (1.00, 1.28)
	≥100 mg/dL	1515 (7.36)	Ref.	Ref.	Ref.	Ref.
≥180 mmHg	<70 mg/dL	325(9.97)	1.16 (1.02, 1.32)	1.15 (1.01, 1.31)	1.16 (1.02, 1.33)	1.14 (0.97, 1.35)
	70-100 mg/dL	617 (8.35)	0.95 (0.86, 1.06)	0.95 (0.86, 1.06)	0.97 (0.87, 1.07)	0.93 (0.81, 1.06)
	≥100 mg/dL	1045 (8.71)	Ref.	Ref.	Ref.	Ref.
*P* for interaction			0.649	0.646	0.608	0.255
In-hospital mortality						
<140 mmHg	<70 mg/dL	51 (2.19)	1.38 (0.98, 1.95)	1.32 (0.93, 1.86)	1.34 (0.95, 1.90)	1.13 (0.72, 1.76)
	70-100 mg/dL	66 (1.53)	0.96 (0.70, 1.32)	0.94 (0.69, 1.30)	0.96 (0.70, 1.32)	0.98 (0.66, 1.46)
	≥100 mg/dL	96 (1.59)	Ref.	Ref.	Ref.	Ref.
140-180 mmHg	<70 mg/dL	128 (2.03)	1.39 (1.13, 1.71)	1.27 (1.03, 1.57)	1.25 (1.01, 1.54)	0.99 (0.76, 1.30)
	70-100 mg/dL	203 (1.53)	1.04 (0.87, 1.25)	0.98 (0.82, 1.17)	0.99 (0.82, 1.18)	0.86 (0.69, 1.08)
	≥100 mg/dL	302 (1.47)	Ref.	Ref.	Ref.	Ref.
≥180 mmHg	<70 mg/dL	117 (3.59)	1.13 (0.92, 1.40)	1.06 (0.86, 1.32)	1.07 (0.87, 1.33)	0.80 (0.61, 1.04)
	70-100 mg/dL	231 (3.13)	0.98 (0.83, 1.16)	0.94 (0.80, 1.11)	0.97 (0.82, 1.14)	0.86 (0.70, 1.06)
	≥100 mg/dL	382 (3.19)	Ref.	Ref.	Ref.	Ref.
*P* for interaction			0.667	0.697	0.715	0.647

Data are OR (95% CI) unless otherwise stated. Model 1 adjusted for age and sex. Model 2 adjusted for variables in model 1 plus body mass index (<25.0 or ≥25.0 kg/m^2^), systolic blood pressure, diastolic blood pressure, smoking status, drinking status, hypertension, diabetes mellitus, previous ICH, medication history (including prior use of antiplatelet, anticoagulant, antihypertensive agent, and stains), and creatinine. Model 3 adjusted for variables in model 2 plus GCS score on admission as a sensitivity analysis.

## Data Availability

Data are available to researchers on request for purpose of reproducing the results or replicating the procedure by directly contacting the corresponding author.

## Supplementary Materials

Supplementary Materials See Table S1 in the Supplementary Material for baseline characteristics between included and excluded ICH patients.
